# Financial Automation Audit Method Based on Blockchain Technology

**DOI:** 10.1155/2022/9941585

**Published:** 2022-07-05

**Authors:** Weidong Gai, Yue Gu, Jiaming Qin

**Affiliations:** ^1^Accounting College, Wuhan College, Wuhan 430022, Hubei, China; ^2^University Bridge (Optical Valley Blockchain) Mass Innovation Space, Wuhan 430022, Hubei, China

## Abstract

Blockchain (BC) maintains a continuously growing database in a “decentralized” way, and its impact on the financial auditing industry is becoming increasingly significant. This paper aims to study the research on financial automation auditing methods supported by blockchain technology and proposes the related concepts of blockchain technology, hash function, financial auditing analysis, and the impact of BP Neural Network (BPNN) and its algorithms on financial automation auditing methods. Simultaneously, this paper likewise disperses the poll overview to definite individuals, for example, endeavor, monetary work force, focus and ranking directors, university researchers, and specialists, who have pragmatic support in the execution and use of monetary review. The experimental results of this paper show that speculation based on the interconnected environment is the most basic natural factor for understanding this idea, and its score is also the largest at 4.36 points.

## 1. Introduction

The rapid development of Internet technology, massive data, cloud computing, artificial intelligence, and massive data chains has had a large impact on the future economic development trend. With its unique advantages, blockchain technology has been widely used in finance, credit, Internet of Things, insurance, and other fields. Blockchain technology can help related industries reduce costs, improve efficiency, and inject new vitality into them. With the vigorous development of digital currencies (such as Bitcoin), increasingly people recognize that blockchain technology is the basic technology that supports the development of various fields.

As of now, there are many imperfections and dangers in the credit component. Blockchain-based dispersed encoded records take care of the issue of absence of credit and essentially affect the present modern climate and plan of action. The disseminated record of the blockchain takes on a brought-together calculation, and in this biological system, the distributed course technique and the Lightning Network can significantly further develop the work efficiency. The dispersed record of the blockchain cannot just enormously work on the security and straightforwardness of information, yet additionally diminish the expense of data procurement.

The innovations of this paper are as follows. (1) The use of blockchain technology to research financial automation audit has certain innovation and practicability. (2) By analyzing the technical characteristics of blockchain, this paper constructs the application framework of blockchain financial auditing and expounds the application advantages of blockchain in financial auditing.

## 2. Related Work

Blockchain is the technology behind the Bitcoin cryptocurrency system; it is considered attractive for ensuring enhanced security and untraceable privacy protection in some implementations for various applications in many other areas such as the Internet of Things (IoT) ecosystem. Currently, academia and industry are conducting in-depth research on the application of blockchain technology in various applications. The purpose of Sikorski's research is to explore the application of blockchain technology in the fourth industrial revolution (Industry 4.0) and describe and discuss the research and application prospects of blockchain technology related to Industry 4.0 [1]. Miraz conducts a survey of recent research articles and project applications to evaluate the implementation of BC enhanced security, identify associated challenges, and propose solutions for BC-enabled enhanced security systems [2]. Blockchain's requirements and guarantees for cryptocurrency, from transaction throughput to security primitives and privacy, do not match the requirements and guarantees of financial technology (FinTech). Ittay explores how blockchain research beyond Bitcoin is bridging these gaps and some of the remaining challenges [3]. Yeoh aims to study key regulatory challenges affecting blockchain innovative distributed technologies in the European Union and the United States. His findings provide support for blockchain technology [4]. O'Dair M research found that blockchain technology could have transformative potential for the music industry related to recorded music and the sustainability of the music business [5]. Engelhardt presents specific examples of the application of blockchain technology in the health sector, involving near term prospects and challenges [6]. The downside of these studies, however, is that the considerations are not comprehensive enough to adapt to more complex situations, and precision needs to be improved.

## 3. Blockchain Technology and Related Methods

### 3.1. Definition and Structure of Blockchain

#### 3.1.1. Definition of Blockchain

Blockchain is a decentralized, collectively maintained, and cryptographically secure distributed database that cannot be tampered with. Through the nodes in the network, the data information in a cycle is stored in a block by cryptographic methods. Then, each block generates a unique hash value as a characteristic value, and then these blocks are connected in a time sequence and a chain structure to form a blockchain. The main characteristics of blockchain include anonymity, decentralization, trustlessness, collective maintenance, and reliable database. Decentralization really intends that there are no extraordinary hubs in the blockchain network, and every hub has similar privileges and commitments. Any node has the right to access the data block list and read the data information in it, each node does not affect others, and the damage of individual nodes will not cause problems to the overall network. Trustless means that because the blockchain is efficient and transparent in the process of recording information and the recording method is very secure, it cannot be tampered with and is difficult to forge, and nodes cannot deceive each other and do not need mutual trust. Collective maintenance means that every node in the entire blockchain can participate in maintenance. Reliable database means that the storage method of the blockchain is distributed storage, and the data can be copied and shared among all network nodes, instead of being made into multiple backups. Any node can download complete data information, and a single node cannot modify the content. Only nodes that control more than 51% can affect the database [7].

According to these characteristics of blockchain, this technology can be used in all application fields that require fairness and honesty, which is why this article chooses blockchain technology. The application of blockchain in this paper belongs to a large medical data operation record book, involving every user in the operation process, as shown in Figure 1. The layers of blockchain technology include data layer, network layer, consensus layer, incentive layer, contract layer, and application layer. Combined with the use of this article, this chapter will introduce the data layer, network layer, consensus layer, and the security of blockchain analysis.

#### 3.1.2. Data Layer

Each block on the blockchain is connected in turn. When a new block appears and is recognized by other nodes, this block will be connected to the previous block chain and form the latest block chain. The blockchain main chain is the longest blockchain in this period from the time of the formation of the founding block to the birth of the current block. It records the complete history of blockchain data, and all data can be traced back to the main chain. However, if two blocks appear at the same time in a short period of time, the main chain of the block will fork. At this time, the block chain will no longer be in consensus and the participants must wait for the appearance of the next block to rebuild the consensus. Blocks need to choose to connect to the blockchain with the largest proof of work, which is the main blockchain, because the way to resolve forks in consensus is for nodes to choose the longest chain [8, 9].

As shown in Figure 2, block A and block B appear at the same time in a short time after block N3, and both A and B meet the conditions. At this time, it is necessary to make a judgment based on the situation after A and B. If block C and other blocks are connected to block B, then the BC chain is the main chain. For attackers, the large amount of generated fake information means that it takes a lot of computing power to find a longer blockchain to replace the current consensus. That is to say, when more than 51% of the computing power is controlled, the famous “51%” attack may occur, but this situation is rare [10].

#### 3.1.3. The Workflow of Blockchain

Figure 3 is a schematic flowchart of the blockchain, and the specific steps are as follows [11].

1. A hub needs to start another information record, and the hub needs to communicate this information record to all hubs in the whole organization through the P2P organization.
2. Other nodes receive the data and store the received data records in the block.
3. The node that generates the block broadcasts its block to all nodes in the entire network.
4. Other nodes verify the broadcasted block. If the block is successfully verified by other nodes, that is, a consensus of the whole network is reached, the block will be added to the main chain of the block. At this time, it needs to go back to step 1 and wait for a new message to be broadcasted.

#### 3.1.4. Key Technologies of Blockchain

Blockchain technology originates from Bitcoin, a peer-to-peer cash system proposed in 2009. Subsequently, Bitcoin was developed in the open source community, and a variety of encrypted digital currencies were evolved based on Bitcoin, which realizes the key technologies used by Bitcoin, including proof-of-work mechanism, Merkle Tree data verification, P2P communication model, digital signature and encryption, and reward mechanism. The blockchain technology stack is shown in Figure 4 [12].

With the in-depth research on blockchain technology, including the multiparty contributions of the open source community, there are now a variety of blockchain technology implementations.

#### 3.1.5. SWOT Analysis Matrix Theory

SWOT analysis matrix is a relatively basic comprehensive information analysis tool. The so-called SWOT refers to the advantages and disadvantages of the enterprise and the opportunities and threats that may exist in the environment of the enterprise. SWOT analysis is essentially a comprehensive and systematic analysis of the company's own situation and development environment [13]. First, analyze the enterprise itself and discover all advantages and disadvantages of the enterprise; second, analyze the development environment in which the enterprise is located, and determine the possible opportunities and threats. Through SWOT analysis, the company's current strategic panorama can be reflected more comprehensively (as shown in Table 1).

SO strategy means that the enterprise chooses a growth strategy; WO strategy is a reverse strategy; ST strategy is a diversification strategy; WT strategy is a defensive strategy.

SWOT matrix analysis is conducive to helping enterprises give full play to their advantages, avoid disadvantages, promote strengths and avoid weaknesses, turn weaknesses into advantages, and turn challenges into opportunities, which is of great significance to helping enterprises formulate future development strategies. In short, the SWOT matrix is a method of comprehensive analysis and comprehensive evaluation of the subject's own conditions and environment.

### 3.2. Hash Function

#### 3.2.1. Definition and Properties of Hash Function

The hash function is to compress messages of any length and finally output a fixed-length hash value [14, 15]. Its mathematical expression is

(1) $$\begin{array}{c} W:{\left\{0,1\right\}}^{*}⟶{\left\{0,1\right\}}^{n},B=W\left(K\right). \end{array}$$

Among them, W represents the adopted hash function, {0,1}^*∗*^ is the message space, {0,1}^*n*^ is the space of the output message digest value, K represents the input message of any length, and B is the final output message digest value.

Hash functions have many practical applications in cryptography. To achieve their functions, they must have the following properties:

1. The length of the message involved in the calculation is arbitrary.
2. The final output value of the function is a fixed length, and the size of the length depends on the specific function.
3. For any known message *K*, it is easy to calculate the value of *W*(*K*).
4. Given the value of B, a message K cannot be found by calculation, so that *B* = *W*(*K*), and this property is also the one-way of the hash function.
5. For any given message K, another message *K*′(*K*′ ≠ *K*) cannot be found by calculation, so that *W*(*K*)=*W*(*K*′). If a one-way hash function satisfies this property, then the hash function is said to satisfy weak collision resistance.
6. It is computationally infeasible to find any two different messages K and *K*′(*K*′ ≠ *K*) that satisfy equation *W*(*K*)=*W*(*K*′). A hash function that satisfies this condition has strong collision resistance.

Among the above six properties, the first three are the basic requirements that the hash function can be used for message authentication, and the last three are the basic security properties of the hash function to meet different applications.

#### 3.2.2. Classic Hash Function

To better research and analyze hash functions, this section will briefly introduce a commonly used hash function SHA1.

The operation process of the SHA1 algorithm is described as follows:

(a) Message stuffing: it produces message packet *B*_1_, *B*_2_,…, *B*_*L*−1_ of length 512XL bits.
(b) Initialize link variables:
  (2) $$\begin{array}{c} A=W_{0}^{0}=0x67452301,\\ B=W_{1}^{0}=0xEFC\;DA\;B89,\\ C=W_{2}^{0}=0x98BA\;DC\;FE,\\ D=W_{3}^{0}=0x10325476,\\ E=W_{4}^{0}=0xC3\;D2E1F0. \end{array}$$
(c) Compressing function processing:
  (3) $$\begin{array}{c} \left\{\begin{array}{cc} M_{t}=K_{t}^{i}, & 0\leq t\leq 15,\\ M_{t}=ROTL^{1}\left(M_{t-3}⊕M_{t-8}⊕M_{t-14}⊕M_{t-16}\right), & 16\leq t\leq 79. \end{array}\right. \end{array}$$
  Among them, *ROTL*^*u*^(*X*) means to rotate *x* to the left by *u* bits. *S*_*t*_ a is an additive constant, each round takes a different value, and its value is expressed as follows: *t* represents the number of rounds of iteration.
  (4) $$\begin{array}{c} \left\{\begin{array}{cc} S_{t}=ox5A82799, & 0\leq t\leq 19,\\ S_{t}=ox6E\;D9EBA1, & 20\leq t\leq 39,\\ S_{t}=ox8F1BBC\;DC\;, & 40\leq t\leq 59,\\ S_{t}=oxCA62C1\;D6, & 60\leq t\leq 79. \end{array}\right. \end{array}$$
(d) It gets the final hash value: in each step function operation, the values in *A*, *B*, *C*, and *D* will be assigned to the *B*, *C*, *D*, and *E* registers in turn. At the same time, the current input values of *A*, *B*, *C*, *D*, *E*, the addition constant, and the value of the message word generated by the message block are operated by the step function, and the obtained value is assigned to the register *A*, and its expression is
  (5) $$\begin{array}{c} \left\{\begin{array}{c} A=\left(ROTL^{5}\left(A\right)+g_{t}\left(B,C,D\right)+E+M_{t}+K_{p}\right)\mathrm{mod}2^{32},\\ B=A,\\ C=ROTL^{30}\left(B\right)\mathrm{mod}2^{32},\\ D=C,\\ E=D. \end{array}\right. \end{array}$$

Among them, *t* is the number of steps, 0 < *t* < 79, *p* is the number of rounds, 1 < *p* < 4, and the calculation formula of *g*_*t*_ is as follows:

(6) $$\begin{array}{c} g_{t}\left(b,c,d\right)=\left(b\wedge c\right)\vee \left(\bar{b}\wedge d\right),0\leq t\leq 19,\\ g_{t}\left(b,c,d\right)=b⊕c⊕d,20\leq t\leq 39,\\ g_{t}\left(b,c,d\right)=\left(b\wedge c\right)\vee \left(b\wedge d\right)\vee \left(c\wedge d\right),40\leq t\leq 59,\\ g_{t}\left(b,c,d\right)=b⊕c⊕d.60\leq t\leq 79. \end{array}$$

After each message block is operated, the obtained value is assigned to the registers *A*, *B*, *C*, *D*, and *E*, the value in the current register is modulo added to the input value of this operation, and the current intermediate link variable value is obtained. When the value of the last message block is calculated sequentially, the obtained value is the final message digest.

### 3.3. Financial Audit

#### 3.3.1. Risks Faced by Auditing under the Conditions of Informatization

Relevant scholars have investigated and analyzed the reasons for informatization auditing and reached the conclusions shown in Table 2 [16]. It also objectively describes the risk factors faced by the audit.

#### 3.3.2. Innovations in the Application of Blockchain Technology to Auditing

The various characteristics of blockchain technology show that this technology is very suitable for application in the audit industry. It can improve and perfect the shortcomings of the traditional audit industry, ensure the quality of accounting information, and greatly liberate the productivity of auditors [17].

1. Improve the efficiency of audit work: (a) the starting point of early audit implementation; (b) the authenticity of audit data; (c) the efficiency of obtaining evidence.
2. Optimize the audit workflow: on the one hand, the basic audit work is intelligentized, which greatly reduces the basic work of auditors. Auditors can devote more energy to more complex work that requires data analysis based on the actual situation. The quality of the audit will be improved, and the results of the audit will be more professional and in depth. On the other hand, auditors no longer need to formulate a detailed and complex audit plan. The audit of most businesses can be realized as early as the moment economic business occurs, and there is no need to wait until the financial report is prepared before auditing.
3. Reduce the cost of audit work.

The innovative diagram of blockchain technology applied to auditing is shown in Figure 5.

#### 3.3.3. The Process of Financial Audit Analysis Model

Audit analysis models can be divided into individual audit analysis models, category audit analysis models, and system audit analysis models according to their functions. Most of the individual audit analysis models are to carry out audit verification and extraction of doubts based on the specific problems of the audited object. The category audit analysis model is to conduct targeted audits on the scope and content of the nodes according to the characteristics of the audited units. The system audit analysis model systematically analyzes the financial status of the audited unit from the overall perspective, studies the overall financial risk level of the audited unit, and provides support for enterprise leaders to make decisions. Among them, the relationship between the three point, line, and plane, and category audit analysis is a specific extension of system audit analysis [18, 19].

Different types of audit analysis models have their own thematic functions. The system audit analysis model is mainly used to grasp the system, the category audit analysis model is mainly used for key locking, and the individual audit analysis model is mainly used for clue screening. The general audit analysis model construction sequence is to first build the system audit analysis model, then the category audit analysis model, and finally the individual audit analysis model. The process of audit analysis model is shown in Figure 6. The types and data sources of intelligent financial reports are shown in Table 3.

#### 3.3.4. Construction of an Intelligent Financial Reporting Model Based on Blockchain Technology

The data needed in the financial report generation process come from various business data, and the specific collection process is shown in Figure 7 [20]. When the economic activity of the enterprise occurs, the financial data submission system will initiate storage and quickly transmit it to the relevant authorized nodes in a point-to-point form. After automatic preprocessing, the accounting transaction data are generated and put into the database, and the legal basis for the integrity verification of transaction information is stored synchronously. Other nodes will wait to query the database for unconfirmed transaction information. Once confirmed, the transaction information can be packaged to form a block code. The authorized node verifies the legitimacy of the transaction through the data processing algorithm and then processes the relevant transaction data and adds the timestamp and other specific identification content and adds it to the new block.

Blockchain technology is a decentralized database management solution, which is fully applied in the process of organizing accounting information. It builds a blockchain-based financial report generation model through decentralized storage and intelligent analysis. The specific process is shown in Figure 8 [21].

### 3.4. BP Neural Network and Its Algorithm

BP (Back Propagation) neural network is a multilayer forward network to tutor learning based on error back propagation algorithm training, and it is composed of multiple neurons connected to each other according to certain criteria. BP Neural Network (BPNN) is essentially the problem of solving the minimum value of the error function, which is an important and classic algorithm [22].

#### 3.4.1. Basic Structure of BP Neural Network

The signal of BPNN is forward conduction. The signal is transmitted from the input node to the hidden layer node through weighting and function transformation, and its value is

(7) $$\begin{array}{c} D_{j}=F\left({\text{net}}_{j}\right)\;,j=1,2,\text{…},m,\\ {\text{net}}_{j}=\sum_{i=0}^{n}U_{ij}G_{i},j=1,2,\text{…},m. \end{array}$$

For the BP network with multihidden layer structure, the signal is transmitted from the hidden layer of the previous layer to the next hidden layer; for the single hidden layer structure shown in the figure, the signal is directly transmitted from the hidden layer to the output layer, as follows:

(8) $$\begin{array}{c} V_{k}=F\left({\text{net}}_{k}\right)\;,j=1,2,\text{…},k,\\ {\text{net}}_{k}=\sum_{j=0}^{m}R_{jk}G_{j}\;,k=1,2,\text{…},s. \end{array}$$

Among them, *F*(*X*) is called the transfer function, and the unipolar sigmoid function (hyperbolic tangent function) is generally used:

(9) $$\begin{array}{c} F\left(B\right)=\frac{1}{1+E^{-X}}. \end{array}$$

Making it differentiable and continuous,

(10) $$\begin{array}{c} F^{\prime }\left(B\right)=F\left(B\right)\left[1-F\left(B\right)\right]. \end{array}$$

Sometimes, depending on the application needs, a bipolar sigmoid function can also be used:

(11) $$\begin{array}{c} F\left(B\right)=\frac{1-E^{-B}}{1+E^{-B}}. \end{array}$$

#### 3.4.2. BP Learning Algorithm

The core idea of the BP learning algorithm is to repeat the forward conduction of error and the reverse conduction of error until the output error meets the design requirements.

The expected output of the neural network is *A*=(*A*_1_, *A*_2_,…, *A*_*l*_)^*T*^, and the output error *e* is defined as

(12) $$\begin{array}{c} e=\frac{1}{2}{\left(A-L\right)}^{2}=\frac{1}{2}{\sum_{k=1}^{s}\left(A_{k}-L_{k}\right)}^{2}. \end{array}$$

Expanding the above formula layer by layer in reverse. For the hidden layer, there are

(13) $$\begin{array}{c} e=\frac{1}{2}\sum_{k=1}^{s}{\left[Y_{k}-F\left({\text{net}}_{k}\right)\right]}^{2}=\frac{1}{2}{\sum_{k=1}^{s}\left[Y_{k}-F\left(\sum_{j=0}^{m}V_{jk}D_{j}\right)\right]}^{2}. \end{array}$$

Expanding further to the output layer, there are

(14) $$\begin{array}{c} e=\frac{1}{2}\sum_{k=1}^{s}{\left\{A_{k}-F\left(\sum_{j=0}^{m}V_{jk}F\left({\text{net}}_{k}\right)\right)\right\}}^{2}=\frac{1}{2}{\sum_{k=1}^{s}\left\{A_{k}-F\left(\sum_{j=0}^{m}V_{jk}F\left(\sum_{i=0}^{n}U_{ij}B_{i}\right)\right)\right\}}^{2}. \end{array}$$

(15) $$\begin{array}{c} \Delta V_{jk}=-\eta \frac{\partial e}{\partial v_{jk}}. \end{array}$$

(16) $$\begin{array}{c} \Delta U_{ij}=-\eta \frac{\partial e}{\partial U_{ij}}. \end{array}$$

In the above two formulas, the constant *η* is the learning rate, which can affect the speed of weight adjustment, which in turn affects the speed of the entire learning process. When *η* ∈ (0,1) and *η* are larger, it is easier to jump out of the local minimum interval of the output error *e*, and the learning speed is faster, but the adjustment accuracy is poor.

Substituting the expression of *E* in (13) and (14) into the gradient adjustment in (15) and (16), the weight adjustment formula of the 3-layer BPNN can be obtained:

(17) $$\begin{array}{c} \Delta V_{jk}=\eta \left(A_{k}-L_{k}\right)L_{k}\left(1-L_{k}\right)D_{j},\\ \Delta U_{ij}=\eta \left(\sum_{k=1}^{s}\left(A_{k}-L_{k}\right)L_{k}\left(1-L_{k}\right)V_{jk}\right)D_{j}\left(1-D_{j}\right)B_{i}. \end{array}$$

The derivative of the unipolar sigmoid function, equation (10), is applied. For multihidden layer BPNN, it is only necessary to reversely derive the weight adjustment formula according to the above rules.

## 4. Experiment of Financial Automation Audit Method Based on Blockchain Technology Support

Agreement system implies that all hubs in the blockchain arrive at a brought-together agreement on the refreshed record data, and the agreement component can completely ensure that the information data are valid and safe. The logical framework of the blockchain application platform is shown in Figure 9.

### 4.1. Questionnaire Results

The study was directed through an electronic study known as the “poll star” and scattered to instructors inside the extent of the brand name through the Internet filling, e-mail, and phone interviews of the review star. It fundamentally incorporates definitive people, for example, corporate money instructors; focus and ranking directors, who have useful cooperation in the execution and utilization of bookkeeping informatization; and university rationale assessment laborers, scientists, and other staff, to guarantee the greatness, authority, and adequacy of the exploration results. After a few rounds of assessment of public sentiment, 255 overviews were actually disseminated, including 20 invalid studies and 235 authentic reviews (as shown in Table 4).

### 4.2. Relevant Information Based on the Questionnaire Survey

According to the results collected by the questionnaire, the relevant issues related to the application of blockchain technology to the accounting information system are analyzed, as shown in the following figure.

Figure 10(a) depicts the results of the respondents' evaluation of the credibility of the current financial automation audit. It can be seen from the figure that the highest proportion of evaluations is less credible, accounting for 41.84% and 51.53% of those who think that they are completely untrustworthy and those who think that they are less credible, accounting for half of the respondents. According to the answers of professionals and authoritative persons, the reliability of financial automation audit is not very good at present, which is a major problem of financial automation audit. Therefore, the research in this paper is meaningful.

Figure 10(b) depicts the respondents' understanding of whether the industry has applied blockchain technology; the figure shows that as much as 53.57% of people are familiar with the industry that uses blockchain technology. Due to the obscure and cutting-edge nature of blockchain technology, most nonprofessionals are unaware of this technology. However, in this questionnaire, as many as half of the professionals are familiar with it, which once again proves the validity of the results of this questionnaire.

### 4.3. Ranking of the Importance of Realizing the Concept of the Credibility Guarantee Mechanism of the Accounting Information System Based on Blockchain Technology

Through the above analysis, we can know that it is necessary and important to build the financial automation audit credibility guarantee mechanism of blockchain technology to a large extent. Therefore, the conditions that should be met to realize this idea, or the difficulties that still need to be overcome, also require further analysis. Next, we made descriptive statistics on the idea of realizing the credibility assurance mechanism of financial automation audit based on blockchain technology. The detailed results are shown in Table 5.

As can be seen from Table 5, the score of each subproject in this project is greater than 4 points, so each project is essential for realizing the concept of the credibility assurance mechanism of financial automation auditing based on blockchain technology. However, the research of this paper is based on the assumption of an interconnected environment, so this condition is also the most basic environmental factor to realize this idea, and its score is also the largest, with a score of 4.36. In addition, it also requires the maturity of related technologies, the reduction of integration costs, and the support of relevant legal systems as support. The scores of these projects are also roughly similar. In today's “Internet +” era, science and technology are developing rapidly, and the IoT is growing rapidly, so the realization of these conditions is just around the corner. Traditional industries need to be integrated with Internet technology in order not to be eliminated by the times and to develop more fully. Therefore, relevant theoretical research is essential and important, and it is also a strong foundation for realizing the idea.

## 5. Discussion

Blockchain technology is a data sequence that arranges data packets into blocks in chronological order, ensuring that the data are not tampered and forged. Therefore, the ledger of the blockchain is decentralized, authoritative, and immutable.

The upsides of evaluating in the blockchain climate mostly lie in the rightness of information assortment. Exchange information is put away in the blockchain, which tackles the ongoing issue of information assortment and capacity and guarantees the security of information stockpiling.

Real-time audit, blockchain real-time audit, and technical characteristics solve the real-time problem in traditional audit. Through the early warning of the application mechanism of the real-time audit platform, the losses caused by the audit unit due to strategic decision mistakes or poor management cannot be recovered.

## 6. Conclusions

This paper sums up the characteristics and advantages of blockchain advancement through a hierarchical overview of blockchain development and a popular assessment study of specialists acquainted with blockchain advancement. Through additional investigation, focusing on the advancement of blockchain, this paper makes a hierarchical examination on the viability of monetary computerization review and the wellbeing, unwavering quality, and adequacy of the affirmation part and observes that the monetary robotization review in light of blockchain innovation can meet the believability necessities.

## Figures and Tables

**Figure 1:** Blockchain technology hierarchy.

**Figure 2:** Schematic diagram of the main chain.

**Figure 3:** Schematic diagram of blockchain process.

**Figure 4:** Blockchain technology stack.

**Figure 5:** Innovation diagram of blockchain technology applied to auditing.

**Figure 6:** Audit analysis model flowchart.

**Figure 7:** Data collection process based on blockchain technology.

**Figure 8:** Financial report generation process based on blockchain technology.

**Figure 9:** Logical framework diagram of the blockchain application platform.

**Figure 10:** Respondents' evaluation of the credibility of financial automation audits and their understanding of blockchain technology. (a) The respondents' evaluation of the reliability of financial automation auditing. (b) The degree of understanding of the respondents about blockchain technology.

**Table 1:** SWOT analysis matrix style.

Strategic choice	Strengths	Weaknesses
Opportunities	SO strategy (growth strategy)	WO strategy (turnaround strategy)
Threats	ST strategy (diversification strategy)	WT strategy (defensive strategy)
Difference	A little	More

**Table 2:** Analysis of reasons for implementing informatization audit.

Reasons for implementation	proportion
Keep up with key controls	25.89%
Rapid response to events	22.61%
Reduce the consumption of audit resources	9.8%
Improve audit efficiency	9.8
Compliance needs	6.7%
Meet timeliness needs	6.0%
Implement the company's financial policies	3.3%
Other	16.3%

**Table 3:** Types of smart financial reports and data sources.

Reporting model	Type of report	Data sources
Economic event based reporting	Sales report, fund raising report, debt report, etc.	Purchase and sale contract, purchase order, receipt and payment, document, delivery, document, payslip, value-added tax bill, investment agreement, debt contract and bank receipt, etc.
Comprehensive income report	Performance report, revenue report	Sales contract, special VAT invoice, bills receivable, receipt voucher, etc.
Interactive on-demand reporting	Information management, business intelligence reporting	Data extraction on demand
Real-time intelligent financial reporting	Automatic multi-dimensional financial reporting	Data extraction on demand
Intelligent analysis report	Internal management, budget implementation, financial performance evaluation, industry comprehensive analysis, etc.	Financial data and business activities, financial indicators and enterprise operation indicators

**Table 4:** Basic information of the questionnaire.

Personnel characteristics	Category	Sample size	Percentage (%)
Work unit category	State-owned enterprise	55	23.40
	Private enterprise	104	44.26
	Government-affiliated institutions	46	19.57
	Other	30	12.77
Industry category	Finance	44	18.72
	Construction	65	27.66
	Service industry	52	22.13
	Manufacturing	26	11.06
	Retail	20	8.51
	Other	28	11.91
Job category of personnel	Financial staff	126	53.61
	Scientific research/education personnel	71	30.21
	Other	38	16.17
Personnel position category	Middle and senior managers	106	76.26
	Financial professional and technical personnel	33	23.74
Personnel age	Under 25	25	10.64
	25–35 years old	139	59.15
	35–45 years old	51	21.70
	Over 45	20	8.51

**Table 5:** Descriptive statistics of the concept of realizing the credibility assurance mechanism of financial automation audit based on blockchain technology.

Specific items	Sample size	Minimum value	Maximum	Mean value	Standard deviation
The Internet plus and the IoT are developing at a high speed and are in an environment of full interconnection.	235	1	5	4.36	.771
The relevant professional technologies supporting this concept are gradually mature and have a realistic basis for realizing the concept.	235	2	5	4.11	.682
The realization of innovative technology can be better connected with traditional technology to minimize the integration cost.	235	1	5	4.29	.755
Regulators need to recognize this concept and need to be bound by relevant systems and laws.	235	2	5	4.33	.677

## Data Availability

Data sharing is not applicable to this article as no datasets were generated or analyzed during the current study.
